The article "Analysis of the Clinical Effect of Music Combined with Hypnosis on Labor Analgesia Based on Data Mining" was retracted in 2023. Reasons: signs of a paper mill; suspected computer-generated content; unreliable results or conclusions; lack of ethics approval or compliance.

# Analysis of the Clinical Effect of Music Combined with Hypnosis on Labor Analgesia Based on Data Mining

**DOI:** 10.1155/2021/1418281

**Published:** 2021-10-15

**Authors:** Jie Chen, Yaer Chen, Fang Wang, Chunbo Qiu

**Affiliations:** Ningbo University Medical School Affiliated Hospital, Ningbo, Zhejiang 315000, China

## Abstract

The objective of this paper is to study the curative effect of music combined with hypnosis on labor pains during childbirth. Based on the algorithm of data mining, we randomly selected 100 women who delivered babies in obstetric units from October 2020 to June 2021, set the control group and the observation group, obtained the relevant clinical data through comparison, and analyzed the value of music combined with hypnotic analgesia midwifery in obstetrics. The results showed that the number of spontaneous delivery cases in the observation group was higher than that in the control group (*P* < 0.05) and the delivery time in the observation group was better than that in the control group (*P* < 0.05). It is proved that music combined with hypnosis can effectively improve the rate of natural childbirth and shorten the overall labor time, so as to guarantee the health of mother and child.

## 1. Introduction

The cesarean section rate in China has always been among the top in the world. Pain stress and psychological stress coexist during childbirth. In particular, primiparous women lack psychological preparation for childbirth and are prone to feel anxiety and fear, which leads to an increase in dystocia and unindicated cesarean section. In order to seek a more effective analgesic delivery method, 100 samples were selected for analysis and study in this study, so as to explore a natural analgesic delivery method without side effects and drug intervention, so as to improve the comfort feeling of pregnant women during delivery, reduce the rate of cesarean section, and reduce the occurrence of adverse outcomes for mother and child [1]. Generally, the depth of hypnosis is divided into three levels: shallow, moderate, and deep. ① In the shallow level, the subject is quiet and relaxed, the muscles of the body are relaxed, and the hands and feet are heavy. The subject maintains a certain degree of judgment and can be aroused by strong external stimuli. ② In the moderate level, the subject shows drowsiness, body muscle relaxation and weakness, suggestive enhancement, and poor judgment [2]. Skin pain is reduced, although the subject can judge but not escape. ③ In the deep level, the subject's facial expression is dull, her muscles are loose, and she only keeps a single line of contact with the hypnotist. She does not feel any stimulation around her, showing high suggestibility and losing self-control and judgment, etc. [3]. We aim to observe the physiological effects of light and moderate hypnotic therapy on parturient and fetal analgesia under the background of music therapy.

The article "Analysis of the Clinical Effect of Music Combined with Hypnosis on Labor Analgesia Based on Data Mining" was retracted in 2023. Reasons: signs of a paper mill; suspected computer-generated content; unreliable results or conclusions; lack of ethics approval or compliance.

Music therapy refers to the systematic intervention of therapists in the treatment process through the use of a variety of different forms of music experience, so as to help patients achieve better treatment results. The three key elements are the music, the therapist, and the object of treatment. Hypnotherapy refers to the use of scientific hypnotherapy technology, so that the patient is put into the hypnotic state, and then the positive suggestion is given to the patient, so as to control the patient's physical and mental state of a psychological therapy. With the research development of the two therapies, music combined with hypnotherapy has gradually developed and then been applied in many fields [4]. It is a comprehensive approach that integrates physiology, psychology, and medicine to broaden the understanding of treatment. The mechanism of music hypnotherapy is to make the music experience compete with the pain experience. The music experience of afferent nerve channel can reduce the pain experience and dilute the pain experience, so as to achieve the effect of pain relief [5]. Hypnotherapy is to change the physical and mental state of the patient in the hypnotic state under the guidance of the therapist, so as to replace the negative thoughts with positive thoughts. Hypnotic analgesia is effective in childbirth, headache, etc. The key is not the type of pain, but the different hypnotic methods used according to the pain [6, 7]. Pain will cause some stress reactions, such as fear, anxiety, and irritability; these reactions stimulate the sympathetic nerve to make it excited, and maternal body will release catecholamine, causing uterine vasoconstriction, which is not conducive to childbirth. Clinically, music and hypnosis can play a certain role in relieving pain. When the human body is in a dormant state, the perception of pain will decrease accordingly, so as to achieve the purpose of analgesia and then help the smooth progress of labor [8–10]. Music is one of the three major factors in music therapy, the choice of which is critical. The specific choice is affected by two aspects: The first is the maternal own feeling toward the music. Due to the differences in aesthetics, taste, and so on, different individuals will have different experience for the same music, so the choice of music is important to ensure that the music is suitable for maternal preferences. The second is the stage of labor. The rhythm of the music can have an effect on the birth process. In the process of childbirth, the choice of relaxed, soft, and regular rhythm of music as far as possible can have a better effect. In the early stage of labor, soothing music helps women relax and calm, and in the active period of labor, music with a slightly stronger sense of rhythm can guide women to exert force regularly, thus speeding up the labor process. For example, the rhythm of music such as “Spring River Flower Moonlight Night” and “Lotus Blooms Everywhere” is close to the human heart rate, neither too fast nor too slow. Its melody and rhythm are more in line with the labor process, which is more suitable for the labor process of music. The volume of music needs to be controlled properly, about 40 to 50 decibels, which can achieve better effects [11]. In conclusion, to ensure the comfort of pregnant women, different music should be selected for each delivery stage. Zhong et al.'s studies have shown that music can effectively reduce the pain of maternal latency and the pain in active period is not obvious. In addition, we have reduced the maternal pain in an active period and the self-hypnosis of the maternal self-hypnosis, and the effect is superior to peer research [12]. The results of this study show that music combined with hypnosis has a better analgesic effect in obstetrics. Hypnosis belongs to the category of psychology. In pregnant women who are 6-7 months pregnant, hypnosis and self hypnosis are necessary. Therefore, it is very important for the selection and training of Hypnotists. In addition, the degree of hypnosis is proportional to the maternal acceptance; it is impossible to have a strong maternal hypnosis, and it is impossible to hypnotize, so the maternal choice is also very critical [13]. The results of Li et al. showed that hypnosis has better analgesic effect. This is close to our findings, but at the same time we also found that shumei ointment, moderate music can help the mother relax, achieving better analgesic effect on hypnosis and simple muscles. We also found that in spite of the effect of pain hypnosis, the environment is also important; noisy environment is not conducive to maternal hypnosis [14]. According to the research data, the severe pain in the latent and active period of pregnant women will increase the incidence of cesarean section and fetal distress and adversely affect maternal and child health [15]. Therefore, using epidural approach is necessary. However, intraspinal administration is often used to relieve pain. According to the data of complications of intraspinal analgesia, almost all analgesics and drugs can cause maternal hypotension, somnolence, nausea and vomiting, dizziness, nerve damage, and weakness of contractions and can also lead to neonatal respiratory depression, heat maternal and neonatal infections, etc.

The article "Analysis of the Clinical Effect of Music Combined with Hypnosis on Labor Analgesia Based on Data Mining" was retracted in 2023. Reasons: signs of a paper mill; suspected computer-generated content; unreliable results or conclusions; lack of ethics approval or compliance.

In 1986, the Internet had its first “congestion crash” when throughput from LBL to UC Berkeley dropped from 32 Kbps to 40 Bps. Subsequently, people proposed four core algorithms of TCP congestion control, namely, slow start, congestion avoidance, fast retransmission, and fast recovery. With the explosive development of the network, these core algorithms are also constantly being improved, and new variants of the slow start algorithm have appeared: smooth start, limited slow start, P-Start, and other improvement methods. A common idea in these improvements is to gradually reduce the growth of the transmission window as the transmission rate approaches the network bandwidth, ensuring a smooth transition to the congestion avoidance phase. Although music and hypnotherapy have been gradually applied in clinical midwifery in China, there is still a lack of certain standards, so it may be difficult for intervention to achieve the expected effect [16]. Maternal cooperation is also very important in the treatment of maternal music therapy object and is one of the three major factors, pregnant women may have negative emotions because of physical pain. At this time, she needs effective guidance and encouragement from medical staff, with music to help her calm down to relieve pressure and anxiety. Therapists are also one of the main factors in music therapy. For various reactions in the delivery process, it is necessary to pay close attention to and deal with them in time and finally complete the delivery process of music therapy. During the whole course of treatment, it is also crucial to choose the appropriate hypnotic guide [17]. Nursing staff assume an extremely heavy task and role. If the level of nursing staff is low, it may be difficult for the treatment to achieve the expected effect, so it is necessary to carry out more professional training for nursing staff, so as to promote the music therapy to play a greater role. Beautiful music can make people feel happy, so as to relieve the pressure and relax the mood. Hypnosis can effectively guide patients into the hypnotic state and then guide their mental and physical relaxation [18, 19].

Based on the existing research, this paper randomly selects 100 pregnant women who delivered in obstetrics from June 6, 2020, to December 2020 based on the data mining algorithm. The parturients were divided into control group and observation group. By comparing the relevant clinical data, the practical value of music combined with hypnotic analgesia in obstetric delivery was analyzed. The results showed that the number of cases of natural delivery in the observation group was higher than that in the control group (*P* < 0.05), and the delivery time in the observation group was better than that in the control group (*P* < 0.05). The analgesic means of music combined with hypnosis can improve the rate of natural childbirth and shorten the whole labor time to ensure the health of mother and child.

The article "Analysis of the Clinical Effect of Music Combined with Hypnosis on Labor Analgesia Based on Data Mining" was retracted in 2023. Reasons: signs of a paper mill; suspected computer-generated content; unreliable results or conclusions; lack of ethics approval or compliance.

## 2. Research Methods

### 2.1. General Information

A total of 100 puerperae who delivered babies in our hospital from October 2020 to June 2021 were selected. All the pregnant women were primiparae, with single child, and aged 19–28 years. Gestational weeks ranged from 35 to 42. Gynecological examination, B-ultrasound examination, and auxiliary examination excluded pelvic stricture, abnormal fetal position, pregnancy hypertension syndrome, and other complications of pregnancy. Prenatal blood routine, electrocardiogram, and liver and kidney function were normal. When the puerperae came to the hospital for obstetric examination, the professional hypnotic midwives trained them in self-hypnosis. Professional hypnotic midwives were selected for participating in hypnotism according to the following criteria: they must have work experience of more than 5 years, rich clinical professional experience, good psychological quality, and 1 month of professional hypnotic training. Finally, 50 cases were selected as the treatment group. The control group included 50 cases of women who did not receive self-hypnosis training or who were not suitable for self-hypnosis training. There was no statistical significance in age, gestational age, measurements outside the pelvis, fetal size estimates, and other general data between the two groups (*P* > 0.05), showing comparability. See Table 1.

### 2.2. Test Methods

Assume that the preset empirical value (or the energy value before the electrode patch falls off) is Presets and that the real-time energy value is CurrEnergy. With reference to previous studies on dark adaptation and based on the thought of the latter stage of P-Start slow start algorithm, the algorithm designed in this paper is shown in Algorithm 1.

The Stanford Hypnotic Sensitivity Scale was used to determine 100 puerperae who were suitable for self-hypnosis training. The specific methods were as follows: patients in the control group were given analgesia under epidural anesthesia, and patients in the treatment group were given analgesia by music combined with hypnosis and midwifery. The specific methods are as follows: on the basis of the application of hypnotic drugs, give the patient music therapy; before the patient delivery, understand the patient's music preferences; in the drug hypnosis, play the patient's favorite music, so that the patient's mood can keep relaxed and happy, into the state of sleep. According to the different labor pain period of the patient, adjust the length of the music, so that the patient's mood keeps relaxed. Pregnant women should be instructed to practice by themselves at home, 15–20 min each time, twice a day, so that hypnosis and self-hypnosis methods can be applied to the whole process of childbirth. The opening of uterus in the treatment group was 3 cm wide, and the pregnant women were taken to the waiting room by professional midwives. The puerperae chose their favorite music, such as smooth rhythm, moderate strength, little fluctuation, and soft music; arrange the puerpera to lie on a comfortable bed for delivery; let her focus on staring at the front of a light, slowly inhale, with chest slightly expanded halfway, exhale through mouth, repeat this several times and relax the muscles of the whole body. After the puerpera entered the self-hypnosis state, the midwife made language suggestions to the puerpera such as “your eyes began to be tired,” “your hands and feet began to relax,” “your whole body has been relaxed,” “you are more and more relaxed,” and “you are energetic, happy” and then further deepened the hypnosis into the deep hypnosis state. Midwives can according to the situation by the self or midwife input corresponding instructions to effectively control muscle movement and induce the disappearance of pain, so that most women in satisfaction and pleasure, through the birth canal, will slowly squeeze the baby out and successfully complete the delivery process. After the delivery, suggestive language was used to awaken the puerpera to complete the whole music hypnotherapy process. The two groups of puerperae could be properly administered static point oxytocin according to the uterine contractions during labor. In the treatment group, there were 20 cases of oxytocin application, with an application rate of 40%; the control group had 45 cases of oxytocin application, with an application rate of 85%; and the difference was statistically significant (*P* < 0.01).

The article "Analysis of the Clinical Effect of Music Combined with Hypnosis on Labor Analgesia Based on Data Mining" was retracted in 2023. Reasons: signs of a paper mill; suspected computer-generated content; unreliable results or conclusions; lack of ethics approval or compliance.

### 2.3. Observation Indicators

Subjective pain was measured by midwives at the first stage of labor latency, the first stage of labor activity, and the second stage of labor. After the delivery, the time of the first stage of labor, the second stage of labor, and the number of cases of natural delivery and cesarean section were statistically summarized. According to the chief complaint pain grading method (VRS), pain is divided into four grades as follows:

  Level 0: no pain.
  Level I: mild pain; the patient has pain, but can endure it, can live a normal life, and can sleep at night.
  Level II: moderate pain; the patient obviously feels pain, cannot tolerate it, cannot sleep at night, and needs to take analgesics.
  Level III: severe pain; the patient feels intense unbearable pain, is unable to sleep at night, and strongly needs to take analgesics.

(1) $$\begin{array}{c} \text{effective rate}=\frac{\left(\text{grade 0}+1\right)}{\text{total number of cases}}\times 100\text{\%.} \end{array}$$

### 2.4. Statistical Analysis

SPSS 13.0 statistical software was used. Measurement data were expressed as *x* ± s *t*-test was used, and counting data were tested by *χ*2 test. *P* < 0.05 was considered statistically significant.

## 3. Research Results

The degree of pain in the treatment group was significantly lighter than that in the control group, and the difference was statistically significant (*P* < 0.01), as shown in Table 2.

The total length of labor in the treatment group was significantly lower than that in the control group, and the difference was statistically significant (*P* < 0.01) (see Table 3).

The rate of cesarean section in the treatment group was significantly lower than that in the control group, and the difference was statistically significant (*P* < 0.05) (see Table 4).

The usage rate of oxytocin in the treatment group was significantly lower than that in the control group, and the difference was statistically significant (*P* < 0.01), as shown in Table 5.

In the experiment, the energy value gradually increases from 0 to Presets according to the above increase. The real-time energy value at each critical moment is shown in Figure 1.

As can be seen from the chart in Figure 1, the increase of the energy output of the analgesic instrument decreases gradually with the increase of the real-time energy value, and the increase process of the real-time energy value is relatively smooth on the whole. The average time of labor in the control group was 8.21 ± 3.12 h, and that in the treatment group was 13.16 ± 5.11 h. The average time of labor in the control group was significantly shorter than that in the treatment group (*P* > 0.05).

Hypnosis using music is a new way of hypnotic analgesia. Combined with music, hypnosis for labor analgesia does not affect the contractions and circulation mechanics, but music can have a positive effect on the patient's central nervous system. Music can reflect people's feelings in real life. When people enjoy music, their mood will also be affected by music. For example, fast music can make people feel excited, sad music can make the listener feel sad, and slow music can make people relax. When patients are clinically guided to give birth, they can relax their nerves by playing gentle and soothing music, so as to actively cooperate with doctors to give birth, so that the level of obstetric treatment is effectively improved.

The article "Analysis of the Clinical Effect of Music Combined with Hypnosis on Labor Analgesia Based on Data Mining" was retracted in 2023. Reasons: signs of a paper mill; suspected computer-generated content; unreliable results or conclusions; lack of ethics approval or compliance.

Music and hypnosis for obstetric analgesia belong to the nondrug therapy in natural childbirth. Music therapy has been widely used in clinical practice and has achieved certain curative effect. Self-hypnosis has achieved good pain relief or even painless effect in natural childbirth and can shorten the labor process at the same time. Music combined with hypnotherapy significantly reduced the degree of pain in uterine contractions, shortened the total length of labor, reduced the rate of cesarean section, increased the rate of natural delivery, and reduced the use rate of oxytocin. Music and hypnosis have a certain effect on reducing pain and speeding up the labor process by improving the factors that hinder labor. Music intervention can effectively shorten the length of the first stage of labor and the second stage of labor, thus speeding up the labor process. Music therapy speeds up the labor process and is able to promote natural labor, which in turn increases the birth rate.

Labor pain is the necessary process of production, in order to minimize the pain of patients, in the process of labor, labor analgesia will be carried out, as it can reduce the pain of labor fear and greatly reduce the rate of cesarean section. The methods of present labor analgesia are mainly divided into drug analgesia and nondrug analgesia. The use of music in hypnosis is a new way of hypnotic analgesia which does not affect the contraction and circulation mechanics, but can positively affect the central nervous system of patients through music.

## 4. Conclusions

In order to study the effect of music combined with hypnosis on puerperae after labor pain, in this paper, based on the data mining algorithm, 100 women who gave birth in obstetric units during June 2020 to December 2020 were randomly selected, and the control group and the observation group were set up. Relevant clinical data were obtained through comparison, and the value of music combined with hypnotic analgesia in obstetric labor was analyzed. The results showed that the number of cases of natural delivery in the observation group was higher than that in the control group (*P* < 0.05), and the delivery time in the observation group was better than that in the control group (*P* < 0.05). The analgesic means of music combined with hypnosis can improve the rate of natural childbirth and shorten the whole labor time to ensure the health of mother and child. In conclusion, through our study, we found that music combined with hypnosis for obstetric analgesia is a simple, easy, economic, safe, and effective way of labor analgesia; has a good development and application prospect; and is worth promoting in hospital obstetric units.

The article "Analysis of the Clinical Effect of Music Combined with Hypnosis on Labor Analgesia Based on Data Mining" was retracted in 2023. Reasons: signs of a paper mill; suspected computer-generated content; unreliable results or conclusions; lack of ethics approval or compliance.

## Figures and Tables

**Figure 1:** Real-time energy curve.

**Algorithm 1:** The algorithm designed in this paper.

**Table 1:** Comparison of basic information of parturient women in the two groups.

Group	Age (years)	Gestational week (weeks)	External pelvic measurement (cm)	Fetal size estimation (g)
The treatment group (*n* = 50)	24 ± 3	38 ± 3	8.3 ± 0.5	3285 ± 215
The control group (*n* = 50)	23 ± 5	38 ± 5	8.4 ± 0.6	3310 ± 185
*T* value	1.5	0.5	1.1	1.0
*P* value	>0.05	>0.05	>0.05	>0.05

**Table 2:** Comparison of pain degree of uterine contractions between the two groups.

Group	Level 0	Level I	Level II	Level III	To be efficient (%)
The treatment group	0	29	19	2	62
The control group	0	16	30	4	30
Total	0	45	49	6	92
*χ*2					34
*P* value					<0.01

**Table 3:** Comparison of duration of labor between the two groups.

Group	The first labor (min)			The second labor (min)		
	120–180	180–240	>240	<60	60–120	>120
The treatment group	43	5	2	46	4	0
The control group	24	25	1	9	39	2
*χ*2		55			84	
*P* value		<0.01			<0.01	

**Table 4:** Comparison of cesarean section rate between the two groups.

Group	Vaginal delivery	Cesarean delivery	Cesarean delivery rate (%)
The treatment group	45	5	8
The control group	42	8	16
*χ*2			6.5
*P* value			<0.05

**Table 5:** The intravenous point of oxytocin in the two groups of women.

Group	Oxytocin used	No oxytocin used	Total	Usage (%)
The treatment group	14	36	50	28
The control group	38	12	50	76
*χ*2				53
*P* value				<0.01

## Data Availability

The data used to support the findings of this study are available from the corresponding author upon request.

## References

[1] Yuanyuan L., Huang H., Weiliang M., Ruohai L., Jun L. (2017). A concentration-response observation of hydromorphone combined with ropivacaine in labor analgesia. *Zhonghua Yixue Zazhi*.

[2] Bombardieri A. M., Wildes T. S., Stevens T., Wolfson M., Avidan M. S. (2019). Practical training of anesthesia clinicians in electroencephalogram-based determination of hypnotic depth of general anesthesia. *Anesthesia & Analgesia*.

[3] Casiglia E., Albertini F., Tikhonoff V. (2018). Experimental approach to the transmission of information in hypnosis. *Psychology*.

[4] Tingyuan Y., Wang E., Cui X., Ju J. (2019). Effects of ropivacaine-sufentanil epidural analgesia on labor and maternal and neonatal outcomes. *Medicinal Plants*.

[5] Keppler J. (2018). Shedding light on the fundamental mechanism underlying hypnotic analgesia. *Annals of Palliative Medicine*.

The article "Analysis of the Clinical Effect of Music Combined with Hypnosis on Labor Analgesia Based on Data Mining" was retracted in 2023. Reasons: signs of a paper mill; suspected computer-generated content; unreliable results or conclusions; lack of ethics approval or compliance.

[6] Belur Nagaraj S., Ramaswamy S. M., Weerink M. A. S., Struys M. M. R. F. (2020). Predicting deep hypnotic state from sleep brain rhythms using deep learning. *Anesthesia & Analgesia*.

[7] Matinella A., Brugnoli M. P., Pasin E., Segatti A., Concon E., Squintani G. (2017). 70. laser-evoked potentials (leps) in chronic pain conditions during hypnotic analgesia. *Clinical Neurophysiology*.

[8] Li C. J., Xia F., Xu S. Q., Shen X. F. (2020). Concerned topics of epidural labor analgesia: labor elongation and maternal pyrexia. *Chinese Medical Journal*.

[9] Rajesh K. S., Rajan L., Kumar (2019). Analgesia%bupivacaine%epidural%fentanyl%labor. *Anesthesia: Essays and Researches*.

[10] Ngan Kee W. D., Ng F. F., Khaw K. S., Tang S. P. Y., Koo A. G. P. (2017). Dose-response curves for intrathecal bupivacaine, levobupivacaine, and ropivacaine given for labor analgesia in nulliparous women. *Regional Anesthesia and Pain Medicine*.

[11] Johnson A. J., Elkins G. R. (2020). Effects of music and relaxation suggestions on experimental pain. *International Journal of Clinical and Experimental Hypnosis*.

[12] Zhong H. Y., Yang Z. Y., Zhang W., Cai S. (2019). Effects of adding oxycodone to ropivacaine on labor analgesia: a randomized controlled trial. *The Clinical Journal of Pain*.

[13] Wang X., Zhang J., Feng K. (2019). The effect of hypothermia during cardiopulmonary bypass on three electro-encephalographic indices assessing analgesia and hypnosis during anesthesia: consciousness index, nociception index, and bispectral index. *Perfusion*.

[14] Li M. J., Wei B. X., Deng Q. X., Liu X., Zhang Y. (2019). Effect of preemptive electroacupuncture on pain reactions in primiparous parturients during vaginal delivery. *Zhen ci yan jiu = Acupuncture research/[Zhongguo yi xue ke xue yuan Yi xue qing bao yan jiu suo bian ji]*.

[15] Farran H. A., Abeer E., Farhat M. D. (2019). The effect of epidural neostigmine combined with levobupivacaine on neuraxial analgesia during labor. *The Medical Journal of Cairo University*.

[16] Morell E., Peralta F. M., Higgins N., Suchar A., Fitzgerald P., McCarthy R. J. (2020). Effect of companion presence on maternal satisfaction during neuraxial cplabor analgesia: a randomized clinical trial. *Obstetric Anesthesia Digest*.

[17] Asgarlou Z., Mohseni M., Khosravizadeh O., Ahmadi S., Moosavi A. (2019). The effects of epinephrine, as a supplement for epidural and spinal anesthesia, on the duration of analgesia during childbirth and apgar score: a systematic review and meta-analysis. *Nursing and Midwifery Studies*.

[18] An F.-P., Liu J.-e., Wang J.-r. (2021). Medical image segmentation algorithm based on positive scaling invariant-self encoding cca. *Biomedical Signal Processing and Control*.

The article "Analysis of the Clinical Effect of Music Combined with Hypnosis on Labor Analgesia Based on Data Mining" was retracted in 2023. Reasons: signs of a paper mill; suspected computer-generated content; unreliable results or conclusions; lack of ethics approval or compliance.

[19] Zuyun, Jiang X., Sun X., Wang X. (2020). Image defogging algorithm based on sky region segmentation and dark channel prior. *Journal of Systems Science & Information*.

